The article "Blocking TRPV1 in Nucleus Accumbens Inhibits Persistent Morphine Conditioned Place Preference Expression in Rats" was retracted in 2020. Reasons: manipulated images; concerns about the images.

# Blocking TRPV1 in Nucleus Accumbens Inhibits Persistent Morphine Conditioned Place Preference Expression in Rats

**DOI:** 10.1371/journal.pone.0104546

**Published:** 2014-08-13

**Authors:** Li-Jun Heng, Bo Huang, Heng Guo, Lian-Ting Ma, Wei-Xin Yuan, Jian Song, Peng Wang, Guo-Zheng Xu, Guo-Dong Gao

**Affiliations:** 1 Department of Neurosurgery, Tangdu Hospital of Fourth Military Medical University, Xi'an, Shaanxi, China; 2 Department of Neurosurgery, Wuhan General Hospital of Guangzhou Military Command, Wuhan, Hubei, China; 3 Department of Neurosurgery, PLA Chengdu General Hospital, Chengdu, Sichuan, China; Universidade do Estado do Rio de Janeiro, Brazil

## Abstract

The function of TRPV1 (transient receptor potential vanilloid subfamily, member 1) in the central nervous system is gradually elucidated. It has been recently proved to be expressed in nucleus accumbens (NAc), a region playing an essential role in mediating opioid craving and taking behaviors. Based on the general role of TRPV1 antagonist in blocking neural over-excitability by both pre- and post-synaptic mechanisms, TRPV1 antagonist capsazepine (CPZ) was tested for its ability to prohibit persistent opioid craving in rats. In the present study, we assessed the expression of TRPV1 in nucleus accumbens and investigated the effect of CPZ in bilateral nucleus accumbens on persistent morphine conditioned place preference (mCPP) in rats. We also evaluated the side-effect of CPZ on activity by comparing cross-beam times between groups. We found that morphine conditioned place preference increased the TRPV1 expression and CPZ attenuated morphine conditioned place preference in a dose-dependent and target–specific manner after both short- and long-term spontaneous withdrawal, reflected by the reduction of the increased time in morphine-paired side. CPZ (10 nM) could induce prolonged and stable inhibition of morphine conditioned place preference expression. More importantly, CPZ did not cause dysfunction of activity in the subjects tested, which indicates the inhibitory effect was not obtained at the sacrifice of regular movement. Collectively, these results indicated that injection of TRPV1 antagonist in nucleus accumbens is capable of attenuating persistent morphine conditioned place preference without affecting normal activity. Thus, TRPV1 antagonist is one of the promising therapeutic drugs for the treatment of opioid addiction.

## Introduction

Opioid addiction is a type of complex brain disorder, which is characterized by uncontrollable opioid craving and compulsive opioid seeking and taking behavior regardless of consequences. High incidence of drug craving and relapse to drug seeking and taking behaviors is the main obstacle for treatment [1]. As traditional therapy fail to work well in preventing relapse in opioid addicts, more effective and target-specific pharmacotherapies with little side effect are in demand.

TRPV1 (transient receptor potential vanilloid subfamily, member 1) is a nonselective cation channel that could be activated by heat, proton, capsaicin and endogenous ligands endovanilloids [2]–[4]. TRPV1 distributed in a variety of areas in the central nervous system [5]–[8]. It has been gradually established that TRPV1 had important role in a series of physiological and pathological status, such as neural development, anxiety and depression. There is still limited information about the function of central TRPV1 in drug addiction, especially in opioid addiction. Previous research suggested that repeated systematic blockade of TRPV1 by capsazepine (CPZ), a TRPV1 antagonist, significantly reduced naloxone-induced withdrawal symptoms [9]. However, there was no further tests of the effect of CPZ on morphine craving or relapse, which is the core process of addiction [1]. Recently, it has been reported that TRPV1 antagonist decreased cocaine-induced cocaine-seeking behavior [10]. Both findings suggest the engagement of TRPV1 in drug addiction behaviors. However, considering the limitation of the animal model used, the difference between opioid and psychostimulant dependence [11] and the peripheral effects accompanying systematic delivery of TRPV1 blocker, further studies are needed to clarify the central action site and behavioral role for TRPV1 in opioid relapse.

Nucleus accumbens (NAc) was known as a critical region in mediating opioid relapse, and has been found to express TRPV1 [5], [6]. Anatomical and electrophysiological studies suggest the possible subcellular localization of NAc TRPV1 is mainly in the presynaptic terminals and the cell bodies [5], [6], [12], [13]. Presynaptic TRPV1 has been proved to facilitate glutamate release and accordingly potentiate glutamatergic transmission in widespread brain areas [13]–[21]. Importantly, the enhancement of glutamatergic synaptic strength via increased presynaptic release in NAc is an essential neuroadaptation during withdrawal associated with opioid dependence [22]. Blockade or attenuation of NAc glutamatergic transmission to reduce the excitatory drive may prevent relapse to opioid use [23]–[25]. In another aspect, TRPV1 present in the cell bodies are proposed to modulate neuronal activity [20]. TRPV1 agonist could increase the spike frequency of neurons in ventral tegmental area [26]. These observations strongly suggested that NAc TRPV1 antagonism might perform anti-relapse effect by limiting neuronal activity and diminishing the efficacy of excitatory inputs from presynaptic terminals, which could reduce morphine conditioned place preference (mCPP) expression [27].

Taken together, the TRPV1 receptor in nucleus accumbens could be a potential target for preventing opioid relapse. In the present study, we test the effect of blocking TRPV1 in NAc on persistent mCPP expression in rats and assess the influence of TRPV1 antagonist on motor activity in the same subjects.

## Materials and Methods

### Subjects and surgery

Male Sprague–Dawley rats (initial weight 200–250 g; Centre of Experimental Animals, Fourth Military Medical University, Xi'an, Shaanxi, China) were individually housed in a temperature- and humidity-controlled vivarium on a 12-hour light/dark cycle. All rats were allowed ad libitum access to food and water. Rats were acclimated to handling daily and allowed to adapt for at least 3 days before the experiment. This study was carried out in strict accordance with the Chinese Animal Welfare Act. The protocol was approved by the Committee on the Ethics of Animal Experiments of Tangdu Hospital of Fourth Military Medical University (Permit Number: TD-5084). All surgery was performed under chloral hydrate anesthesia, and all efforts were made to minimize suffering.

Rats were anesthetized with chloral hydrate (400 mg/kg, i.p.) and implanted with cannulas (0.67 mm of external diameter; Rewardsales, Shenzhen, Guangdong, China) positioned 1.5 mm above each target. The coordinates (Paxinos and Watson, 2005) were as follows respectively: NAc core: anteroposterior (AP), +1.5 mm and mediolateral (ML), ±1.6 mm from bregma; dorsoventral (DV), −6.0 mm from the skull surface; Dorsal striatum (DS): AP, +0.9 mm; ML, ±3.4 mm; DV, −3.8 mm. The cannulas were anchored to the skull with stainless steel screws and dental cement. A stainless steel probe with a plastic cap was inserted into each cannula to keep them unblocked and prevent infection. Rats were allowed to recover from surgery for at least 5d before morphine conditioned preference training. Food intake and body weights were assessed before and after the surgery.

### Morphine conditioned place preference

All experiments were performed in a dimly lit room. The CPP apparatus is composed of two equally sized wooden chambers(25.3×20.1×20.3 cm) separated by a guillotine door. The two chambers differ in their color and floor texture to provide distinct contexts that were paired with morphine or saline injections. One chamber consisted of white walls and a smooth PVC-covered floor with hollow tranverse lines. The other chamber had black walls and a coarse PVC-covered floor with hollow longitudinal lines. The procedure consisted of three different phases: preconditioning test (day 1), conditioning (day 2-day 6), and postconditioning tests, as indicated in Results. In the preconditioning test, each rat was placed in the white compartment with the door open to allow the animal to freely explore the apparatus for 15 min. Animals showing a strong unconditioned preference (>540 s in any chamber), which were 7 of the 135 rats totally used, were discarded. In the subsequent 5 days, conditioning was conducted using a counterbalanced protocol, such that one-half of the animals in each experimental group were conditioned to the spontaneously preferred side and the other half to the spontaneously nonpreferred side. In each conditioning day, the animals received an injection of either morphine (1 mg/kg, 3 mg/kg, 10 mg/kg, s.c.) or saline (1 ml/kg, s.c.) at 9:00–9:30 and were confined for 45 min in the assigned chamber before returning to their home cages. Six hours later, the animals received an injection of vehicle solution (saline, 1 ml/kg, s.c.) and were confined to the alternative chamber for 45 min. In the postconditioning phase, the expression of CPP was tested in withdrawal day 1, 7 (1 w, short-term withdrawal), 14 (2 w) and 21 (3 w, long-term withdrawal) after the last training session. The postconditioning test consisted of placing the animal into the white chamber and allowing it to freely access both chambers for 15 min. Videos of all 15 min tests were captured online and analyzed offline. The amount of time that the animals spend in the conditioned chamber was recorded as CPP score (in seconds).

### Intra-NAc application of CPZ

All rats firstly received mCPP training with 10 mg/kg morphine as described earlier. CPZ was dissolved in DMSO and stored at the concentration of 100 µM, which was diluted to different concentrations for intracranial injection with at most 0.1% DMSO in final solution. Vehicle solutions were prepared accordingly. CPZ (0.1 nM, 1 nM, 10 nM) or vehicle was injected bilateral intra-NAc daily from 3 days before the mCPP expression test during short-term (1 w) or long-term (3 w) withdrawal. CPZ (1 µl) was delivered over 3 min for each side of target. The CPP test was performed 30 min after the last CPZ injection. Furthermore, to examine the target specific effect of CPZ on mCPP, CPZ (10 nM) was injected unilateral NAc or bilateral DS before mCPP test during short-term (1 w) withdrawal.

### Motor activity assessment

To assess the effects of CPZ on motor activity, crossline times were counted manually from the video of mCPP test after CPZ injection. Crossline times was defined as sum of the counts of the subject moving cross the two putative transverse lines trisecting each chamber and the counts of the subject crossing the guillotine door.

### Immunoelectron microscopy

After the behavior test, rats were anesthetized with chloral hydrate (400 mg/kg, i.p.) and perfused intracardially with 100 ml of physiological saline (0.9% NaCl), followed by perfusion with a fixative containing 0.05% glutaraldehyde, 4% paraformaldehyde and 15% picric acid. The brain was removed from the skull and post-fixed in the above fixative without glutaraldehyde at room temperature for 2 hours. Vibratome sections 50 µm in thickness were cut from the blocks. Following washing in 0.01 M PBS, the sections were cryoprotected in 30% sucrose until they sunk. The sections were washed in 0.01 M PBS and incubated in blocking solution (5% NGS+5% BSA) at room temperature for 3 hours. After washing in 0.01 M PBS, the sections were incubated in rabbit anti-TRPV1 antibodies (1∶150, Santa Cruz Biotechnology) and containing 1% BSA for 48 hours at 4°C. Following incubation with the primary antiserum, the sections were processed for immunogold labeling of rabbit TRPV1 antiserum. The tissue was rinsed in PBS and incubated overnight at 4°C in a 1∶50 dilution of colloidal gold conjugated to goat anti-rabbit IgG (Nanoprobes) in 1% BSA. The sections were rinsed in PBS and post-fixed in 2% glutaraldehyde for 45 minutes. They were then rinsed in deionized water 10 times, and the gold particles were silver intensified by a 9-minute incubation in an HQ Silver silver enhancer (Nanoprobes). After rinsing in deionized water and 0.1 M PB 6 times, the sections were osmicated (0.5% OsO4, 1 hour, room temperature), dehydrated and embedded in Durcupan. After examination by light microscopy, the areas of interest were re-embedded and ultrathin-sectioned for electron microscopy. Ultrathin serial sections were collected on formvar-coated single slot grids, stained with lead citrate and washed in distilled water. Sections were observed under an electron microscope (JEM-1230).

The quantity of the symmetric and asymmetric synapses established by TRPV1-positive axon terminals was examined in the NAc. Serial ultrathin sections were made from a depth of ∼3 µm from the surface of the vibratome sections. Every 8th section the TRPV1-stained terminals were analyzed in order, following the rules of systematic random sampling, to avoid sampling the same axon terminals. The number of TRPV1 terminals forming symmetric and asymmetric synapses was calculated for each group and normalized to 3000 µm^2^ to quantify the exact changes in the number of stained terminals in each group. To assess any changes occurring in the density of TRPV1 per terminal, the number of gold particles located in the membrane of the axon terminals was counted and normalized to 1 µm of the terminal's perimeter. Image-Pro Plus 6.0 was used to make the above measurements.

### Western blot

After sacrifice, the brain was dissected, chilled on a glass plate on ice and then cut into slices. The trace of the entry needle was checked to confirm the injection site. According to Atlas of The Rat Brain by George Paxinos & Charles Watson, the area of Bregma ±1.6 mm was removed from the slices and cut limited tissue of NAc, and homogenized in ice-cold homogenizing buffer (50 mM Tris-Cl, pH 7.4, 150 mM NaCl, 5 mM EDTA, 0.1% SDS, 1% NP-40, 1% deoxycholate, 1% Triton X-100, 10 mM PMSF, 50 mM sodium vanadate and 0.1% protease inhibitors cock-tail (Roche, Switzerland)). After centrifugation at 12,000×g for 15 min at 4 °C, the supernatant was collected and the protein content was subsequently assayed by using a BCA Protein Assay Kit (Pierce, Rockford, IL, USA). Equal quantities of total protein (75 µg per lane) were separated by sodium dodecyl sulfate-polyacrylamide gel electrophoresis (SDS-PAGE), followed by transfer to nitrocellulose membranes. The membranes were incubated in 5% milk at room temperature for 2 h. Blots were then incubated with rabbit polyclonal antibody against TRPV1 (1∶1000, Santa Cruz Biotechnology), or β-actin (1∶2000). After washing with buffer, the blots were incubated in anti-rabbit (Zhong Shan, Beijing, China, 1∶1000) secondary antibody conjugated with horseradish peroxide in TBS-T with 5% milk at 4 °C overnight. The blots were visualized using a West Pico Chemiluminescent Kit (Pierce, Rockford, IL, USA), and the density of protein bands quantified by transmittance densitometry using volume integration with LumiAnalyst Image Analysis software.

### Histology

At the end of the behavioral experiments, rats were anesthetized with chloral hydrate (400 mg/kg, i.p.) and perfused intracardially with 10% PBS-buffered formalin. The brains were removed, post-fixed overnight in a 30% sucrose/formalin solution, and then cryoprotected in 30% sucrose/saline. To verify the location of the cannula tips, 40 µm coronal sections were cut through the targeted area (NAc or DS), and stained with cresyl violet, and examined under a light microscope. Rats with off-target cannula placements in only one side of Nac were involved in the Uni-off Nac group for analyses. Rats with incorrect cannula placements were excluded from the study. Overall, six rats were excluded for this reason.

### Data analysis

Data were expressed as Mean ±SEM. Statistical analyses were performed using repeated measures analysis of variance (ANOVA) followed by Duncan *post hoc* tests for multiple comparisons. The accepted level of statistical significance is *p*<0.05.

## Results

### Food intake and body weight after surgery

As shown in Table.1, the daily food intake of surgery animals was similar with control group after the surgery under anesthetized with chloral hydrate. All animals showed increasing body weight after 5-day raise. There were not significant differences of both initial and recovering body weight between control and surgery groups.

**Table 1:** The food intake and body weight of animals after surgery (Means±SEM).

Measured parameters	Control	Surgery
Food intake (g/d)	23.01±4.93	22.76±4.09
Initial body weight (g)	208.96±10.07	211.10±11.28
Body weight after recover (g)	219.92±7.16*	221.20±9.51*

*p<0.05, compared to the initial body weight.

### Morphine conditioned place preference

Higher mCPP scores were observed in morphine conditioned groups (Fig.1). In 1 mg/kg and 3 mg/kg morphine groups, the mCPP expression was numerically increased, but this difference was not significant (F = 0.375, *p* = 0.960). However, comparing to control group, significantly higher mCPP scores in all the 4 postconditioning tests performed at 1 d, 1 w, 2 w, 3 w after last training session were observed in high-dose (10 mg/kg) morphine conditioned group (F = 8.144, *p* = 0.006). There was no significant difference for mCPP score among four time point of postconditioning tests in 10 mg/kg morphine group (*p*>0.05), which indicated that morphine with 10 mg/kg induced a persistent and relatively stable mCPP expression. We chose 10 mg/kg morphine for conditioning training in the CPZ-intervening experiments.

**Figure 1:** Repeated morphine conditioning induced persistent conditioned place preference (CPP) during withdrawal. Morphine conditioned place preference scores (time spent in drug-paired chamber) increased during morphine withdrawal. Sustained increase of mCPP score during morphine withdrawal occurred in high-dose morphine group (10 mg/kg) but not in low- (1 mg/kg) or moderate-dose (3 mg/kg) groups (n = 3). *p<0.01, *vs* SAL group. SAL, saline; MOR, morphine.

### Morphine increased TRPV1 expression in NAc meurons

Levels of TRPV1 in the nucleus accumbens were detected by Western blot and quantitatively analyzed (Fig. 2). Control group revealed the moderate expression of TRPV1 in the nucleus accumbens. There were not significant changes of TRPV1 expression in 1 mg/kg and 3 mg/kg morphine treated groups. However, TRPV1 immunoreactivity was increased markedly in 10 mg/kg morphine withdrawal animals compared with the control group (F = 79.288, *p*<0.01). There were not significant differences of TRPV1 immunoreactivity between 1 week and 3 week morphine withdrawal groups (*p*>0.05).

**Figure 2:** Analysis of western blot results of TRPV1 expression in the nucleus accumbens (NAc). (A) Representative blots of TRPV1. β-actin showed similar protein loading in each group. (B) Densitometric analyses of TRPV1 expression in NAc. The changes were expressed as the ratio to β-actin. Data represent Mean±SEM (n = 3), *p<0.01, *vs* control group.

### Increased TRPV1 located in asymmetric synapses

Transmission electron microscopy was used to examine the expression of TRPV1 in synapse. The immunogold-positive axon terminals were found in both asymmetric synapses (excitatory-type) and symmetric synapses (inhibitory-type) (Fig. 3,Peters et al., 1991).

**Figure 3:** Quantitative changes in TRPV1 expression at the ultrastructural level in morphine withdrawal groups. High-power electron micrographs from the NAc of different groups showing TRPV1 immunogold labeling in the axon terminals forming asymmetric, excitatory-type synapses (A) and symmetric, inhibitory-type synapses (B). In the morphine withdrawal groups the number of gold particles on terminals forming asymmetric synapses increased (A). Graph (C) shows changes in the average number of TRPV1-positive asymmetric and symmetric synapses in each group. The number of TRPV1-positive asymmetric synapses in the morphine withdrawal groups was significantly higher than the control group. However, no difference was found in the normalized number of TRPV1-positive symmetric synapses among all groups. The number of TRPV1-positive symmetric synapses of control were 4.72±0.77, 4.72±0.47 and 4.74±1.00 for 1 d, 1 w and 3 w group respectively. The number of TRPV1-positive asymmetric synapses of control were 7.74±1.38, 7.75±0.77 and 7.74±1.28 for 1 d, 1 w and 3 w group respectively. Graph (D) shows the normalized number of gold particles in TRPV1-positive asymmetric and symmetric synapses. No difference appeared in the normalized number of gold particles in TRPV1-positive symmetric synapses. In contrast, a significant increase occurred in the normalized number of gold particles in TRPV1-positive asymmetric synapses of morphine withdrawal groups versus control group. The normalized number of gold particles in TRPV1-positive symmetric synapses of control were 0.68±0.17, 0.68±0.03 and 0.69±0.04 for 1 d, 1 w and 3 w group respectively. The normalized number of gold particles in TRPV1-positive asymmetric synapses of control were 0.78±0.07, 0.79±0.13 and 0.79±0.03 for 1 d, 1 w and 3 w group respectively. Scale: 200 nm. Data represent Mean±SEM (n = 3), *p<0.05, *vs* control group.

Two vibratome sections from each of three rats in each group were calculated for the absolute number of TRPV1 positive asymmetric and symmetric synapses, and each vibratome section was normalized to 3000 µm^2^. Compared to the control group, a significant increase was found in the number of TRPV1 positive asymmetric synapses in the morphine withdrawal groups (Fig.3C, F = 75.321, *p*<0.05), but no significant change was found in the number of TRPV1 positive symmetric synapses in morphine withdrawal groups (Fig.3C, *p* = 0.622).

To quantify the changes in the number of immunogold particles in certain terminals of the NAc of rats, the number of gold particles in the membranes of TRPV1 stained axon terminals forming symmetric or asymmetric synapses was counted and normalized to the unit perimeter (1 µm) of the axon terminal membrane. Significant increase was observed in the number of immunogold particles in axon terminals forming asymmetric synapses between the control group and morphine withdrawal groups (Fig.3D, F = 36.547, *p*<0.05). In contrast, the number of immunogold particles showed no difference in axon terminals forming symmetric synapses between the control group and morphine withdrawal groups (Fig.3D, *p* = 0.056).

### Intra-NAc CPZ decreased persistent mCPP expression in a target specific manner

To determine whether NAc endovanilloid receptor TRPV1 is involved in the expression of mCPP, rats were given bilaterally repeated intra-NAc injections of different doses of TRPV1 antagonist CPZ during morphine withdrawal. When CPZ was applied during short-term morphine withdrawal, as shown in Fig. 4A, both 1 nM and 10 nM of CPZ significantly decreased mCPP expression at 1 w test (CPZ 1 nM, 370.9±20.2 s; CPZ 10 nM, 371.9±32.5 s; vehicle, 562.0±28.9 s; F = 12.28, *p*<0.01) (Fig. 4A). but the inhibitory effect of 1 nM CPZ was completely eliminated when tested at 3 w with the mCPP score reverted similar to control level (CPZ 1 nM, 522.6±26.4 s; vehicle, 523.3±22.5 s; *p*>0.05) (Fig. 4A). However, the inhibition of 10 nM CPZ could last to 3 w after morphine withdrawal (CPZ 10 nM, 426.8±23.2 s; vehicle, 523.3±22.5 s; *p*<0.05) (Fig. 4A). No active effect of low dose of CPZ (0.1 nM) was observed when tested at 1 w (*p*>0.05) (Fig. 4A). We used higher dose (1 nM or 10 nM) of CPZ for experiments during long-term (3 w) withdrawal. After three times injection, significant inhibition of mCPP expression was observed in both dose of CPZ (CPZ 1 nM, 418.4±19.9 s; CPZ 10 nM, 430.9±26.9 s; vehicle, 505.1±24.6 s; F = 14.86, *p*<0.05) (Fig. 4B). Thus, blocking TRPV1 in NAc disrupts the mCPP expression in both short- and long-term withdrawal. Figure 5 showed the Distribution of infusion sites in nucleus accumbens core.

**Figure 4:** TRPV1 antagonist CPZ administered in bilateral NAc core decreased persistent morphine CPP after both short-(1 w) and long-term(3 w) withdrawal. (A) Dose-dependent effect of CPZ on persistent mCPP expression. Repeated high-dose CPZ (10 nM) injection during short-term morphine withdrawal could induce a complete and prolonged inhibition on mCPP expression. The moderate-dose CPZ (1 nM) has similar but temporary prohibiting effect on mCPP expression, as it could only be observed at 1 w but not 3 w of morphine withdrawal. The low-dose CPZ (0.1 nM) has no influence on mCPP. The upper schedule panel shows the rats were trained conditioned to morphine and received repeated CPZ injections in NAc core after short-term(1 w) withdrawal (n = 11 of Vehicle and CPZ 0.1 nM group, n = 10 of CPZ 1 nM group, and n = 9 of CPZ 10 nM group). (B) CPZ (1 nM and 10 nM) administration eliminated mCPP (n = 7). The upper schedule panel shows the rats were conditioned to morphine and received CPZ injections in NAc core after long-term(3 w) withdrawal. *p<0.01, *vs* control group; ^#^ *p*<0.05, *vs* control group. MOR, morphine; Veh, vehicle; CPZ, capsazepine; NAc, nucleus accumbens.

**Figure 5:** Distribution of infusion sites in nucleus accumbens core. (A) Photograph of representative cannula placements. The cannulas are implanted 1.5 mm above the target. (B) Schematic representations of vehicle or capsazepine injection sites in nucleus accumbens core at the labeled coronal planes. The numbers are the coordinates anterior (+) to bregma in millimeters according to Paxinos and Watson (2005).

To investigate whether CPZ inhibition on mCPP is a target-specific effect, we applied CPZ (10 nM) randomly in unilateral NAc, or bilateral DS during short-term (1 w) morphine withdrawal. Data from rats initially prepared for the bilateral CPZ administration study but with off-NAc cannula placements in only one side confirmed with staining was also analyzed here. As depicted in Figure 6A, in Uni-NAc group, no alteration of mCPP was detected after CPZ injection (CPZ, 549.1±29.7 s; vehicle, 539.0±15.9 s; F = 0.245, *p* = 0.959). Similarly, CPZ injection did not decrease mCPP in the Uni-off NAc group (Fig. 6A). Furthermore, when we examined the CPZ effect on mCPP in the target outside NAc, we found the effective dose of CPZ (10 nM) in DS failed to influence the persistent mCPP expession (F = 0.261, *p* = 0.853) (Fig. 6B).

**Figure 6:** Injection of TRPV1 antagonist CPZ in unilateral of NAc or DS did not change persistent mCPP expression after short-term(1 w) withdrawal. (A) Unilateral NAc CPZ injection (10 nM) or one side off-target during bilateral NAc CPZ infusion (1 nM or 10 nM) failed to affect the sustained mCPP. The upper panel shows the scheme for morphine conditioning, CPZ treatment and mCPP test. Values are Mean ±SEM (n = 7 of Vehicle and Uni-NAc+CPZ group and n = 3 of Uni-off NAc+CPZ group). (B) CPZ (10 nM) injection in DS failed to influence persistent morphine CPP. The upper panel shows rats were conditioned to morphine and received CPZ injections in bilateral DS after short-term withdrawal. Values are mean ±SEM (n = 6 of DS-Vehicle group and n = 7 of DS-CPZ 10 nM group). MOR, morphine; Veh, vehicle; CPZ, capsazepine; NAc, nucleus accumbens; Uni, unilateral; DS, dorsal striatum.

To assess the possible effect of intra-NAc CPZ on motor activity, which could indirectly influence mCPP expression, crossline times of the rats during mCPP tests were analyzed. As shown in Fig.7, there was no statistical difference (*F* = 1.13, *p*>0.05) in crossline times among all groups after CPZ injection in both short-term (1 w) and long-term (3 w) withdrawal. The results confirmed that the alteration of all parameters in the mCPP expression test did not result from changes in motor abilities of rats.

**Figure 7:** TRPV1 antagonist CPZ administered in bilateral NAc fail to affect normal activity after both short-(1 w) and long-term(3 w) withdrawal. (A) All doses of CPZ tested failed to influence the activity of animal measured by photobeam breaks during the 15-min mCPP test (n = 11 of Vehicle and CPZ 0.1 nM group, n = 10 of CPZ 1 nM group, and n = 9 of CPZ 10 nM group). The upper schedule panel shows the rats were trained conditioned to morphine and received repeated CPZ injections in NAc core after short-term (1 w) withdrawal. (B) Both effective doses of CPZ (1 nM and 10 nM) in eliminating sustained mCPP expression fail to affect activity (n = 7). The upper schedule panel shows the rats were conditioned to morphine and received CPZ injections in NAc core after long-term (3 w) withdrawal.Values are mean ±SEM. MOR, morphine; Veh, vehicle; CPZ, capsazepine; NAc, nucleus accumbens.

## Discussion

It is suggested that the NAc glutamatergic system is a key candidate for mediating morphine withdrawal-related addictive behaviors [28], [29]. Alcantara et al. reported that morphine treatment increase the number of synapses of NAc, which was due primarily to an increase in the number of asymmetric synapses, and Asymmetric synapses in the accumbens are characteristic of glutamatergic synapses formed by inputs from other area such as prefrontal cortex, hippocampus and so on [30]. In the present study, we demonstrated that TRPV1 was increased in the nucleus accumbens of rats after morphine conditioned. Significant increase was observed in the number of immunogold particles in axon terminals forming asymmetric synapses between the control group and morphine withdrawal groups. In contrast, it showed no difference in axon terminals forming symmetric synapses, which suggested that the TRPV1 expression at asymmetric synapses might involve in morphine induced CPP. Antagonism of TRPV1 by the selective TRPV1 antagonist CPZ suppressed persistent mCPP expression in rats either during short-term or long-term morphine withdrawal. This inhibitory effect is target-specific, unique for NAc. Conversely, effective doses of CPZ in NAc did not cause significant side-effect on motor activity of the subjects, suggesting the decrease of mCPP expression is not due to motor inhibitory properties of TRPV1 antagonist. Collectively, these results not only extend our understanding on the role of central TRPV1 in drug addiction, but also indicate that TRPV1 antagonist may be a promising type of medication for inhibiting morphine conditioned behaviour.

### Morphine withdrawal increased TRPV1 expression in NAc meurons

TRPV1 is a calcium-permeable cation channel [31], [32]. In the central nervous system, TRPV1 is widely expressed in brain regions including postsynaptic dendrite spines, cell somata [33], and in various layers of the cortex [6], [34]. Previous studies suggested that activation of postsynaptic TRPV1 channels triggered long-term depression in the NAc [12]. Activation of TRPV1 receptors is coupled to glutamate release, which in turn affects the release of GABA, dopamine, and other catecholamines [35], [36]. Activation of TRPV1 in the ventral tegmental area caused excitation of dopaminergic neurons and increased dopamine release in NAc after a painful stimulus [26]. AMPA receptors and GABAA receptors activation are associated with facilitation of motivated behaviors [37].

In the present study, we found that morphine with 10 mg/kg induced persistent and relatively stable mCPP expression lasting from short-term (1 w) to long-term (3 w) withdrawal, which dose has been continuously confirmed to induce sustained mCPP expression in rodents [38], [39]. Accordingly, the expression of TRPV1 in the NAcc was elevated in morphine conditioned animals and maintained in high levels after 1 w and 3 w withdrawal compared to the control group. The increased TRPV1 distributed on the presynaptic membrane of asymmetric synapses. The results indicated that increasing expression of TRPV1 on the presynaptic membrane of asymmetric synapses in NAcc might play an important role in morphine conditioned place preference.

### Intra-NAc CPZ reduced mCPP expression

To confirm the role of TRPV1 in morphine induced conditioned place preference, we injected TRPV1 antagonist CPZ intra-NAc and found that blocking TRPV1 in NAc disrupts the mCPP expression in both short- and long-term withdrawal. Previous study has shown that repeated systematic administration of CPZ could reduce naloxone-induced acute withdrawal symptoms in mice [9]. These findings together reveal the important role of TRPV1 in both psychological and physical aspects of opioid-related behaviors.

At least two possible mechanisms may underlie the inhibitory behavioral effect of TRPV1 antagonist in NAc on mCPP. Firstly, blockade of TRPV1 in NAc may prevent it from overdrive by excitatory inputs essential for CPP. Previous studies have shown that potentiation of glutamatergic inputs on NAc medium spiny neurons is a critical type of neuroadaptation happened during prolonged opioid withdrawal and is associated with relapse [22], [24], [40]. Furthermore, fully or partially blockade of glutamatergic inputs has been proved to disrupt reinstatement to opioid seeking and taking behaviors [23]–[25], [40]. It has been proved that TRPV1 activation facilitate presynaptic neurotransmitter release in variety of brain regions [3], [13]–[17], [19]–[21] and the existence of TRPV1 mRNA in main glutamatergic areas innervating NAc [7]. In the present study, significant increase of the number of TRPV1 positive asymmetric synapses was observed and more immunogold particles in axon terminals in the morphine conditioned rats, which suggested that the inhibitory effect of TRPV1 antagonist on synaptic efficacy should be taken into account when evaluating its inhibitory effect on CPP. Supporting this idea, our finding that the time window for the effectiveness of NAc TRPV1 antagonist on mCPP persisting from short- to long-term drug withdrawal overlapped with the period for NAc glutamate inputs potentiation reported before [22], [41]. Secondly, reduction of NAc neuronal activity by TRPV1 antagonist may also contribute to its effect on mCPP expression. Wu et al [22] reported the increase of intrinsic excitability in NAc neurons during opioid withdrawal, which suggested an enhanced response capability of these neurons. In agreement with these data, increased NAc immediate early gene expression during opioid withdrawal and reinstatement supports the upregulation of NAc neural reactivity during withdrawal [42], [43]. Conversely, blocking NAc activity could reduce mCPP expression and prevent opioid relapse [27]. As is shown previously, membrane depolarization and increase of spiking are essential manifestations after central TRPV1 activation [20], [26], which is mediated by its modulatory on K^+^ and Ca^2+^ conductance or direct Ca^2+^ and Na^+^ influx via the channel itself. Accordingly, blockade of NAc TRPV1, may contribute to limit neural activity in this region, which was confirmed to have relapse-preventing effect [27]. Further studies are necessary to elucidate the above and other mechanisms involved in the action of central, especially NAc, TRPV1 antagonism on drug addiction.

### Intra-NAc CPZ administration did not affect on motor activity

Our data showed that the effective dose of NAc CPZ in preventing mCPP expression failed to influence the locomotor activity. Consistent with previous studies [44], [45], we showed together that this dose range of CPZ is not sufficient to produce behavioral effect on general activity in rats when given alone. However, stimulation of TRPV1 by application of its ligand externally has been shown to suppress spontaneous activity in rodents [15], [45]–[47]. Moreover, blockade of TRPV1 by CPZ has been proved to attenuate hypolocomotor effect of anandamide [47], [48], a ligand for both cannabinoid receptor and TRPV1, which revealed that anandamide induced activity disruption is caused by a TRPV1-dependent mechanism. Collectively, these findings indicate that targeting central TRPV1 may modulate activity of the subject. Nevertheless, discrepancies between these findings and our result implicated that blocking TRPV1 by endogenous ligands in the brain, at least in NAc, may not be sufficient to affect activity, in another word, tonic TRPV1 activation in NAc isn't involved in regulating basal activity. The finding that TRPV1 gene knockout mice showed normal locomotor activity further supports this viewpoint [12]. Thus, blocking TRPV1 in NAc will result in non-effect on activity and the inhibition of CPZ on prolonged mCPP expression is not due to its influence on moving ability of the rats.

In conclusion, the present study indicated the importance of TRPV1 in the NAc in morphine addiction. The increased expression of TRPV1 in the presynaptic membranes of asymmetric synapses in NAc during morphine withdrawal may be one of the mechanisms of mCPP expression. We further demonstrated the inhibitory effect of NAc TRPV1 antagonism on prolonged mCPP expression, which confirmed the involvement of NAc TRPV1 in persistent opioid addiction. Our results support for further mechanism assessment and developing novel treatment targeting central, especially NAc, TRPV1 for mCPP prevention.
